# Research on Energy Supply System Applied to Autonomous Underwater Observation Vehicles

**DOI:** 10.1155/2022/3859307

**Published:** 2022-06-29

**Authors:** Chunjie Wang, Yugeng Chai, Lin Cui

**Affiliations:** ^1^School of Electrical Engineering and Automation, Tianjin University of Technology, Tianjin 300382, China; ^2^Tianjin Complex System Control Theory and Application Key Laboratory, Tianjin 300382, China; ^3^National Ocean Technology Center, Tianjin 300112, China

## Abstract

The discharge characteristics of seawater batteries can be used to prolong the working hours of autonomous underwater observation vehicles. However, the output voltage level of the seawater battery is low, so it cannot directly be used to power supply underwater observation vehicles. In this paper, a boost converter is proposed based on the seawater batteries to power supply autonomous underwater observation vehicles. The proposed converter greatly increases the voltage level of the seawater battery and directly supplies the underwater observation vehicles. Compared with the traditional boost converter, the voltage gain of the proposed converter is more than ten times higher than it under the same duty ratio condition. Its structure is asymmetric interleaved parallel, which can enable power devices to obtain lower voltage stress and ensure that the input current ripple is low. The operating principle and homeostasis property of the proposed converter are analyzed in detail. Finally, a prototype is built. Through simulation and experiment, the correctness of the theoretical design is verified and experimental results are analyzed.

## 1. Introduction

With the improvement of people's understanding of the ocean, the exploration and development of Marine environments covering 70% of the surface has received extensive attention. Autonomous underwater observation vehicle is an autonomous underwater equipment suitable for various environments, characterized by long working hours and wide range of activities [1–6]. Therefore, the energy supply requirements of this equipment are relatively high. Lithium battery has the characteristics of high specific energy and long cycle life [7], began to be applied to the power system of underwater vehicles in the early 21st century [8–11]. However, with the extension of the working hours of autonomous underwater observation vehicle, limited by the volume and weight of the vehicle itself [12–15], lithium battery cannot meet its requirements. Dissolved oxygen seawater battery, with seawater as the electrolyte, carbonized fibre or graphite are used to cathode, and active metal as anode, redox reactions with dissolved oxygen in seawater [16]. The reaction principle is as follows:

Anodes:

(1) $$\begin{array}{c} \text{Mg}⟶{\text{Mg}}^{2+}+2{\text{e}}^{-} \end{array}$$

Cathode:

(2) $$\begin{array}{c} {\text{O}}_{2}+2{\text{H}}_{2}\text{O}+4{\text{e}}^{-}⟶4\text{O}{\text{H}}^{-} \end{array}$$

The output voltage is 1.2-1.4 V, and the battery has an open structure and does not need to design a water pressure shell, which is conducive to generate electricity in seawater at different depths. Compared with lithium batteries, seawater batteries do not need to carry electrolyte and cathode active substance, and the specific energy (318 W h/kg) is higher than lithium batteries (160 Wh/kg) [17–20], and they have the characteristics of long discharge time (3-5 years), safe, and reliable. Therefore, it is particularly suitable for powering equipment that has been working under the sea for a long time. However, due to the low concentration of dissolved oxygen in the ocean, the output power of dissolved oxygen seawater batteries is low [21, 22], and it can only be applied to low-power underwater observation systems of vehicles. Based on the characteristics of the two types of batteries, the energy supply system of autonomous underwater observation vehicle can be designed as shown in Figure 1, lithium battery supplies power the power system of the vehicle, and dissolved oxygen seawater battery supplies power the observation system of the vehicles. Because the power supply technology of lithium battery is relatively mature, it will not be mentioned here.

The output voltage level of dissolved oxygen seawater battery is low, with a rated output of 1.3 V [23], and the voltage level required for observation system is high, so a high-gain DC-DC converter needs to be added to the output side of the seawater battery. The traditional boost converter voltage gain is lower; the higher voltage gain will make the duty cycle close to 1, while power device voltage stress is higher. So the researchers studied how to improve the voltage gain of the converter. Literature [24–26] introduces switched inductors in the boost converter, which increases the voltage gain, but the effect is insufficient. In literature [27, 28], interleaved parallel and switched capacitor are adopted to achieve high gain; due to absence of coupled inductors, the voltage gain of the converter is limited, and the voltage stress of the MOSFET and diode is high. In literature [29], multiset switched capacitors are proposed to obtain high-gain converter, but the increase in the number of switched capacitors undoubtedly increases the cost of circuits, and the efficiency and reliability of the converter cannot be satisfied. In literature [30, 31], coupled inductor was used to achieve high-gain conversion; due to the absence of interleaved parallel, the increase in voltage gain is still limited.

In this paper, a high-gain DC-DC converter with asymmetric interleaved parallel as a framework is proposed, combined with coupled inductor and switched capacitor structure. Firstly, while the converter obtains a higher voltage gain, the voltage stress obtained by the power device is less. On the other hand, the input current ripple of the converter can effectively be suppressed by asymmetric interleaved parallel structure, thus making the seawater battery power supply system more stable. Finally, a prototype is built to verify the feasibility of the proposed converter.

## 2. Principles of Operation and Analysis

The equivalent topology of the proposed converter is shown in Figure 2. The two MOSFET in the converter are controlled by the controller to realize 180° interleaved conduction; the diodes *D*_2_ and *D*_3_ and capacitors *C*_2_ and *C*_3_ constitute the switch capacitor structure and the output diode *D*_4_ as the output of the converter. The input of the converter is a dual coupled inductor structure, including leakage inductance *L*_k1_ and *L*_k2_, magnetizing inductance *L*_m1_ and *L*_m2_, and two ideal transformers; the diode *D*_1_ and the capacitor *C*_1_ form the clamping circuit. The turn ratio of the two coupled inductors can be expressed as *N*_*S*1_/*N*_*p*1_ = *N*_1_ and *N*_*S*2_/*N*_*p*2_ = *N*_2_.

In order to facilitate analysis, it is assumed that the effects of all parasitic elements are ignored. During a cycle, there are 8 working modes and the driving signals of *S*_1_ and *S*_2_ are interleaved 180°.  Figure 3 shows the key waveforms of the proposed converter, and the transient modes I, II, V, and VI due to leakage should be ignored. After ignoring, the modes in a cycle are III, VI, VII, and VIII. The topological stages of the circuit are shown in Figure 4.

In mode III [*t*_2_ − *t*_3_], at *t*_2_, MOSFET *S*_2_ is off, *S*_1_ is still open, diodes *D*_1_ and *D*_3_ are on, and diodes *D*_2_ and *D*_4_ are off, as shown in Figure 4(a). The current on the diode *D*_3_ is expressed as

(3) $$\begin{array}{c} i_{\text{D}3}\left(t\right)=i_{\text{D}3}\left(t_{2}\right)+\frac{V_{\text{C}3}}{n^{2}\left(L_{\text{k}1}+L_{\text{k}2}\right)}\left(t-t_{2}\right). \end{array}$$

In mode VI [*t*_5_ − *t*_6_], at *t*_5_, MOSFETs *S*_1_ and S_2_ are in conduction state, and diodes *D*_1_, *D*_2_, *D*_3_, and *D*_4_ are cut off, as shown in Figure 4(b). The magnetizing inductance *L*_m1_ current is expressed as

(4) $$\begin{array}{c} i_{L\text{m}1}\left(t\right)=i_{L\text{m}1}\left(t_{5}\right)+\frac{V_{\text{in}}}{L_{\text{m}1}+L_{\text{k}1}}\left(t-t_{5}\right). \end{array}$$

In mode VII [*t*_6_ − *t*_7_], at time *t*_6_, MOSFET *S*_1_ is off, *S*_2_ is on, diodes *D*_2_ and *D*_4_ are on, and diodes *D*_1_ and *D*_3_ are off, as shown in Figure 4(c). Input current is expressed as

(5) $$\begin{array}{c} i_{\text{in}}\left(t\right)=i_{\text{in}}\left(t_{6}\right)+\left[\frac{\left(V_{\text{C}1}+V_{\text{C}2}+V_{\text{C}3}+V_{\text{o}}\right)-V_{\text{in}}}{L_{\text{k}1}+L_{\text{m}1}}+\frac{V_{\text{in}}}{L_{\text{k}2}+L_{\text{m}2}}\right]\left(t-t_{6}\right). \end{array}$$

In mode VIII [*t*_7_ − *t*_8_], at *t*_7_, the switch *S*_1_ is kept off, *S*_2_ remains on, diode *D*_2_ is on, and diodes *D*_1_, *D*_3_, and *D*_4_ are cut off, as shown in Figure 4(d). The energy of leakage inductance *L*_k1_ is completely transferred to capacitor *C*_2_, and the current *i*_*S*2_ is expressed as

(6) $$\begin{array}{c} i_{\text{S}2}\left(t\right)=i_{L\text{m}1}\left(t\right)+i_{L\text{m}2}\left(t\right). \end{array}$$

## 3. Performance Analysis

### 3.1. Steady-State and Performance Analysis

According to magnetism chain conservation, the relationship between magnetizing inductance *L*_m1_ and *L*_m2_ is expressed as

(7) $$\begin{array}{c} \left\{\begin{array}{c} Du_{L\text{m}1-\text{on}}+\left(1-D\right)u_{L\text{m}1-\text{off}}=0,\\ Du_{L\text{m}2-\text{on}}+\left(1-D\right)u_{L\text{m}2-\text{off}}=0. \end{array}\right. \end{array}$$

In the formula, *D* is the duty ratio of the *S*_1_ and *S*_2_.

Available in formula (7),

(8) $$\begin{array}{c} V_{\text{C}1}=\frac{V_{\text{in}}}{1-D},\\ V_{\text{C}2}=N_{2}k_{2}V_{\text{in}}+N_{1}k_{1}V_{\text{in}}\frac{D}{1-D},\\ V_{\text{C}3}=N_{1}k_{1}V_{\text{in}}+N_{2}k_{2}V_{\text{in}}\frac{D}{1-D}. \end{array}$$

According to mode VII, the output voltage is expressed as

(9) $$\begin{array}{c} V_{\text{o}}=V_{\text{C}1}+V_{\text{C}2}+V_{\text{C}3}+\frac{V_{\text{in}}}{1-D}. \end{array}$$

The voltage gain is expressed as

(10) $$\begin{array}{c} M_{\text{CCM}}=\frac{2+k_{1}N_{1}+k_{2}N_{2}}{1-D}. \end{array}$$

In the actual coupling inductance design, because the coefficient of coupling is close to 1, it has little effect on the voltage gain. In order to facilitate the analysis, the leakage inductance is not considered in the following case, that is, *k*_1_ = *k*_2_ = 1. The ideal voltage gain is expressed as

(11) $$\begin{array}{c} M_{\text{CCM}}=\frac{2+N_{1}+N_{2}}{1-D}. \end{array}$$

According to formula (11), the ideal voltage gain of the converter is related to turn ratio *n* and the duty ratio *D*. As shown in Figure 5, when *D* remains unchanged, the higher *n*, the higher the voltage gain of the converter.

The voltage stress pushed to *S*_1_ and *S*_2_ is expressed as

(12) $$\begin{array}{c} V_{\text{S}2}=V_{\text{C}1}=\frac{V_{\text{in}}}{1-D}=\frac{V_{o}}{2+N_{1}+N_{2}},\\ V_{\text{S}1}=\frac{V_{\text{in}}}{1-D}=\frac{V_{\text{o}}}{2+N_{1}+N_{2}}. \end{array}$$

The voltage stress of the diode *D*_1_ is expressed as

(13) $$\begin{array}{c} V_{\text{D}1}=V_{o}-V_{\text{C}2}-V_{\text{C}3}=\frac{2V_{\text{in}}}{1-D}. \end{array}$$

The voltage stress of the diode *D*_4_ is expressed as

(14) $$\begin{array}{c} V_{\text{D}4}=V_{\text{o}}-V_{\text{C}2}-V_{\text{C}3}-V_{\text{C}1}=\frac{V_{\text{in}}}{1-D}. \end{array}$$

The voltage stress of the diodes *D*_2_ and *D*_3_ is expressed as

(15) $$\begin{array}{c} V_{\text{D}2}=V_{\text{D}3}=V_{\text{C}2}+V_{\text{C}3}=\frac{N_{1}+N_{2}}{1-D}V_{\text{in}}. \end{array}$$

The ratio curve in Figure 6 is obtained using the ratio *V*_stress_/*V*_o_. It is not difficult to see that the voltage stress of all power devices is lower than output voltage. MOSFETs *S*_1_ and *S*_2_ and diodes *D*_1_ and *D*_4_ decrease with the increase of turn ratio *n*, and diodes *D*_2_ and *D*_3_ increase with it.

### 3.2. Comparison

The high-gain converter is proposed in this paper, fewer power devices are required, and their voltage stress is lower. To further reflect its advantage, the proposed converter is compared with many typical topologies in recent years. The performance parameters are shown in Table 1.

In order to compare the performance of converter, set the coupled inductor turn ratio *n* = 3. The voltage gain comparison curve between the proposed converter and the other four converters is shown in Figure 7, and the proposed converter has a highest voltage gain compared with other typical of boost converters.

The voltage stress comparison curve of the MOSFET is shown in Figure 8. The ratio curve is obtained using the ratio *V*_stress_/*V*_o_. Compared with other typical converters, the proposed converter has the lowest voltage stress, so MOSFET devices with lower voltage stress can be selected at work. Devices with low voltage stress will get smaller loss.

## 4. Design Considerations

### 4.1. Coupled Inductor Design

The turn ratio of the coupled inductor is determined by the voltage gain and the duty ratio, expressed as follows:

(16) $$\begin{array}{c} n=\frac{V_{\text{o}}\left(1-D\right)}{2V_{\text{in}}}-1. \end{array}$$

The value of magnetizing inductance depends on the acceptability of current ripple on the inductance. At the same time, due to the limitations of the characteristics of the seawater cell, the input current ripple large will lead to the unstable output voltage of the seawater cell. Therefore, the coupled inductor current ripple of the converter is set as *α*%. The value of magnetizing inductance is expressed as

(17) $$\begin{array}{c} L_{\text{m}}=L_{\text{m}1}=L_{\text{m}2}=\frac{V_{\text{in}}D}{\alpha \%I_{\text{in}}f_{\text{s}}}=\frac{D\left(1-D\right)V_{\text{o}}}{2\alpha \%I_{\text{in}}f_{\text{s}}}. \end{array}$$

Magnetizing inductance has a great effect on suppressing current ripple, and the input current ripple coefficient under different magnetizing inductance can be obtained, as shown in Figure 9:

The current ripple of the coupled inductor will directly affect the stability of the system. Therefore, according to Figure 9, magnetizing inductance value of 7 *μ*H can be selected to suppress the current ripple and improve the stability of the system.

### 4.2. Capacitor Design

The capacitance is designed based on the voltage ripple and the output power, and the voltage ripple coefficient is *μ*%. The value of *C*_1_ to *C*_4_ is expressed as follows:

(18) $$\begin{array}{c} C_{1}\geq \frac{2P_{\text{o}}}{\mu \%V_{\text{C}1}V_{\text{o}}f_{\text{s}}}=\frac{2P_{\text{o}}\left(1-D\right)}{\mu \%V_{\text{C}1}f_{\text{s}}V_{\text{in}}\left(2n+2\right)},\\ C_{2}\geq \frac{P_{\text{o}}}{\mu \%V_{\text{C}2}V_{\text{o}}f_{\text{s}}}=\frac{P_{\text{o}}\left(1-D\right)}{\mu \%V_{\text{C}2}f_{\text{s}}V_{\text{in}}\left(2n+2\right)},\\ C_{3}\geq \frac{P_{\text{o}}}{\mu \%V_{\text{C}3}V_{\text{o}}f_{\text{s}}}=\frac{P_{\text{o}}\left(1-D\right)}{\mu \%V_{\text{C}3}f_{\text{s}}V_{\text{in}}\left(2n+2\right)},\\ C_{4}\geq \frac{P_{\text{o}}}{\mu \%V_{\text{C}4}V_{\text{o}}f_{\text{s}}}=\frac{P_{\text{o}}\left(1-D\right)}{\mu \%V_{\text{C}4}f_{\text{s}}V_{\text{in}}\left(2n+2\right)}. \end{array}$$

According to the above calculation, based on the actual, the capacitance values of *C*_1_ to *C*_4_ can be the same; in order to make the supply system operate stably, considering the actual circuit parasitic elements, it is necessary to add a certain margin on the basis of theoretical calculation.

The theoretical values and the experiment values of each capacitance can be expressed in Table 2:

## 5. Simulation and Experimental Validation

The designed high-gain converter has a rated power of 10 W and a rated output voltage of 24 V. Seawater battery rated output voltage is 1.3 V. In order to verify the correctness of the above theoretical analysis, the system can be built as shown in Figure 10:

### 5.1. Effect of Simulation Parameters on Current Ripple

In order to further study the working characteristics of the converter, the optimal duty ratio and turn ratio are obtained by simulation. The input current ripple is related to duty ratio and turn ratio. When other device parameters are kept unchanged, the duty ratio of the converter and the turn ratio of the coupled inductor are changed, and the simulation results are shown in Figure 11.

- The current ripple is when *n* = 3, *D* = 50%, the input current
- The current ripple is when *n* = 2, *D* = 60%, the input current
- The current ripple is when *n* = 4, *D* = 40%, the input current

According to formula (17), when the duty ratio increases, the output voltage is kept unchanged, and the current ripple will change with the duty ratio. Therefore, through simulation, the optimal combination of turn ratio and duty ratio in Table 3 can be obtained. When the duty ratio is 50%, the current ripple is the lowest.

After simulation analysis and theoretical analysis, in order to minimize the input current ripple of the system, the coupled inductor turn ratio can be set at 1 : 3. The duty ratio is *D* = 50%.

### 5.2. Simulation Verification

According to the theoretical calculation and the above simulation conclusions, the simulation parameters of Table 4 are set, and the model can be built. The simulation results are as follows.

The simulation waveform of output voltage and *S*_1_, *S*_2_ voltage is shown in Figure 12. The output voltage is 24 V, as shown in Figure 12(a) and the voltage stress of switches *S*_1_, *S*_2_ is 3.8 V, as shown in Figure 12(b). Figures 13 and 14 show the diode voltage simulation waveform, diode *D*_1_ voltage stress is 5.7 V, as shown in Figure 13(a). The voltage stress of diodes *D*_2_ and *D*_3_ is 17.8 V, and diode *D*4 voltage stress is 3.4 V. Current simulation waveform is shown in Figure 15 and the input current ripple value is 0.15 A.

In order to fully verify the performance of the power supply system of the seawater battery under the condition of the proposed converter, the output voltage range (1.2-1.4 V) of the seawater battery is simulated. The simulation results are shown in Table 5:

After simulation, it can be obtained that under the condition that the output voltage range (1.2-1.4 V) of the seawater battery, the input current ripple of the proposed converter is maintained at 0.15-0.29 A, the current ripple is generally low, the voltage stress of the switching device is maintained at 3.54-3.76 V, and the voltage stress is low and the fluctuation is small.

### 5.3. Experiment and Results Analysis

In order to further verify the correctness of theoretical analysis and simulation parameters, a prototype is built in the laboratory, and the experimental waveform is obtained and analyzed.

As shown in Figure 16(a), the load voltage of the converter is about 24 V, which achieves the high gain effect of theoretical analysis. The voltage stress of the MOSFETs *S*_1_ and *S*_2_ is about 4 V. Due to the influence of the parasitic capacitance in the MOSFET, the parasitic capacitance discharge generates the spike voltage shown in Figure 16(b). Because the diode retains a safety margin for the voltage during the selection process, it has little impact on the system. The voltage stress of each diode is shown in Figure 17, the voltage stress of the diode *D*_1_ is about 6 V, *D*_4_ is about 4 V, and *D*_3_ is about 18 V compared to the actual voltage of the diode which is low compared to the theoretical analysis, but the voltage waveform meets the theoretical analysis and has good performance.  Figure 18 is the input current ripple waveform of the converter. Due to the existence of parasitic inductance and parasitic resistance in the actual circuit, the current ripple is somewhat disturbed. It can be seen from the waveform that the current ripple is about 0.2 A, so the structure effectively reduces the input current ripple.

Other output voltage of seawater batteries is tested. Within the output voltage range of seawater batteries, the performance of the 1.2-1.4 V seawater battery power supply system is shown in Table 6.

Through the experimental results, it can be obtained that under the condition of the output voltage of the seawater battery, the current ripple range of the converter is 0.2-0.38 A, and the actual current ripple is close to the simulated current ripple. The influence of parasitic elements in the actual circuit is considered, and the range of current ripples is acceptable. The voltage stress of the switches is 3.67-4 V, compared with the simulation results, and the results are acceptable. The efficiency of the seawater battery power supply system has reached 78.2-84.2%.

### 5.4. Loss Analysis

The main loss in the converter comes from the heating of the power device, where the power device is the coupled inductor, diode, and MOSFET.

#### 5.4.1. MOSFET Loss

The on-state loss of the MOSFET mainly comes from the on resistance *R*_d(on)_ of the switches. The on-state loss is expressed as follows:

(19) $$\begin{array}{c} P_{\text{loss}\left(\text{on}\right)}=R_{\text{d}\left(\text{on}\right)}\times i_{\text{ds}}^{2}. \end{array}$$

In formula (19), *i*_ds_ is the effective value of the current flowing through the DS of the MOSFET.

The shutdown loss of the MOSFETs is not only related to the frequency *f*_s_ but also related to the parasitic output capacitance *C*_oss1_; the shutdown loss is expressed as follows:

(20) $$\begin{array}{c} P_{\text{loss}\left(\text{off}\right)}=\frac{i_{\text{ds}}^{2}\times t_{f}^{2}\times f_{\text{s}}}{48\times C_{\text{oss}1}}. \end{array}$$

The *t*_f_ is the fall time of the switches.

The switching status of the MOSFETs *S*_1_ and *S*_2_ is the same, and the total loss of the switches can be expressed as

(21) $$\begin{array}{c} P_{S}=2\left(P_{\text{loss}-\text{on}}+P_{\text{loss}-\text{off}}\right). \end{array}$$

#### 5.4.2. Diode Loss

The loss on diode is the product of current *i*_F_ and the forward voltage drop *V*_F_ of diode. The loss of diode can be expressed as

(22) $$\begin{array}{c} P_{D}=f_{\text{s}}\times \int_{0}^{T_{\text{S}}/2}V_{F}\times i_{F}\left(t\right)dt. \end{array}$$

#### 5.4.3. Transformer Loss

Transformer loss is the main part of the magnetic component loss. It mainly includes core loss and winding loss, among which core loss includes hysteresis loss and eddy current loss.

The hysteresis loss is proportional to B and is expressed as follows:

(23) $$\begin{array}{c} P_{h}=K_{h}\times f_{\text{s}}\times B^{1.6}\times V. \end{array}$$

*K*_*h*_ is the proportional coefficient related to the material.

The eddy current loss in dynamic alternating magnetic field is

(24) $$\begin{array}{c} P_{c}=\frac{\pi^{2}f_{\text{s}}^{2}B^{2}d^{2}}{6\rho }. \end{array}$$

In formula (24), *d* is the material density, measured in unit g/cm^3^, and *ρ* is resistivity.

Core loss of the transformer may be expressed as

(25) $$\begin{array}{c} P_{\text{core}}=P_{h}+P_{c}. \end{array}$$

Winding loss mainly comes from the copper loss of the primary winding and the secondary winding, which is expressed as *P*_cu_p_ and *P*_cu_s_, including the alternating current winding *R*_ac_p_ and *R*_ac_s_. The *i*_p_, *i*_s_ is the current flowing through, and the losses of the primary side and secondary side winding are expressed as

(26) $$\begin{array}{c} P_{\text{cu}\_\text{p}}=i_{\text{p}}^{2}\times R_{\text{ac}\_\text{p}},\\ P_{\text{cu}\_\text{s}}=i_{\text{s}}^{2}\times R_{\text{ac}\_\text{s}}. \end{array}$$

The winding loss of a transformer is the sum of the copper loss of the primary and secondary side transformers, which is expressed as follows:

(27) $$\begin{array}{c} P_{\text{cu}}=P_{\text{cu}\_\text{p}}+{\text{P}}_{{\text{cu}}_{\text{s}}.} \end{array}$$

The total transformer loss can therefore be expressed as

(28) $$\begin{array}{c} P_{T}=2\left(P_{\text{cu}}+P_{\text{core}}\right) \end{array}$$

#### 5.4.4. Converter Loss Distribution

In fact, there are some other losses in the converter, such as wire loss and delay loss, but these losses are often very small and negligible. After calculation, the loss of each power device is shown in Table 7.

The total power loss of the proposed converter can be expressed as

(29) $$\begin{array}{c} P_{\text{loss}}=P_{S}+P_{D}+P_{T}. \end{array}$$

The loss of each power device is calculated according to the theory, and percentages are reflected in Figure 19. The proportion of transformer loss is the largest. According to the loss analysis, winding loss (*P*_cu_) is considered to be the main loss of the transformer, which is caused by the low rated power of the converter and the high carry currents of the transformer.

Under the rated state of the converter, the ideal conversion efficiency of the proposed converter can be calculated from (29), with a result of 83.1%, and the difference is 1.9% compared with the actual conversion efficiency. Due to the existence of parasitic resistance in the line and the existence of the parasitic capacitance and the parasitic diode in the switching, it has a certain impact on the efficiency of the converter, but the impact is small, and the actual value is close to the theoretical value.

## 6. Conclusions

In this paper, the DC/DC converter in the energy supply system of the autonomous underwater observation vehicles is taken as the research object, exploring the improvement of output voltage level of seawater batteries, through DC/DC converters, to supply power in the underwater observation vehicle. The topology of the proposed converter is studied and verified by simulation and experiment. The main conclusions are as follows:

1. Under the range of output voltage 1.2-1.4 V of dissolved oxygen seawater battery, DC/DC converters can improve the voltage level. Under the premise of maintaining the output voltage of 24 V, the efficiency reaches 78-84%
2. Under the asymmetric interleaved parallel structure, combined with the coupled inductor and clamping circuit, not only the input current ripple is suppressed, but also the voltage stress of the MOSFETs is controlled by about 4 V
3. In the study of improving the voltage level, the combination of coupled inductors and switched capacitance in the topology can enable the converter to obtain higher voltage gain under low duty cycle

## 7. Future Work

Based on the current theoretical calculation and experimental results, an experimental platform for mixed power supply of seawater batteries and lithium batteries will be built. Due to the large loss of transformers in the proposed converter, it will be further optimized to improve the efficiency of the seawater battery power supply system. Further verify the correctness of the proposed system.

## Figures and Tables

**Figure 1:** Energy supply system for autonomous underwater observation vehicles.

**Figure 2:** Equivalent topology of the proposed converter.

**Figure 3:** Key waveforms of the proposed converter.

**Figure 4:** Operation modes of the proposed converter.

**Figure 5:** Voltage gain curve (*N*_1_ = *N*_2_ = *n*).

**Figure 6:** Normalized semiconductor voltage stress versus turn ratios.

**Figure 7:** Comparison of the voltage gain when *n* = 3. (i) Converter in [24, 27]. (ii) Converter in [29]. (iii) Converter in [30]. (iv) Proposed converter.

**Figure 8:** Voltage stress comparison of MOSFET. (i) Converter in [24]. (ii) Converter in [27]. (iii) Converter in [29]. (iv) Converter in [30]. (v) Proposed converter.

**Figure 9:** The relationship between the original inductor and current ripple.

**Figure 10:** Control strategy for the seawater battery.

**Figure 11:** Input current ripple under different duty ratio and turn number ratio.

**Figure 12:** Voltage simulation waveform.

**Figure 13:** Diode *D*_1_ (a) and *D*_2_ (b) voltage waveform.

**Figure 14:** Diode *D*_3_ (a) and *D*_4_ (b) voltage waveform.

**Figure 15:** Input current ripple waveform.

**Figure 16:** Stress wave form of input/output voltage and switches voltage.

**Figure 17:** Diode voltage stress waveform.

**Figure 18:** Input current ripple.

**Figure 19:** Loss distribution of the converter.

**Table 1:** Comparison of the proposed converter to typical converters.

Topologies	No. of switches/diode/capacitors/inductance	Voltage gain	Switch voltage stress
Ref. [24]	1/5/4/2	4/1 − *D*	*V*_o_/2
Ref. [27]	2/4/4/2	4/1 − *D*	*V*_o_/4
Ref. [29]	4/6/6/1	2*n*/1 − *D*	*V*_o_/2*n*
Ref. [30]	1/3/4/2	*n* + 2/1 − *D*	*V*_o_/*n* + 2
Proposed	2/4/4/2	2*n* + 2/1 − *D*	*V*_o_/2*n* + 2

**Table 2:** Comparison of capacitance theory and actual values.

Capacitor	*C*_1_	*C*_2_	*C*_3_	*C*_4_
Theoretical value (*μ*F)	20	60	60	50
Experiment value (*μ*F)	100	100	100	100
Theoretical pressure resistance (V)	6	17.6	17.6	24
Experimental pressure resistance (V)	50	50	50	50

**Table 3:** Input current ripple coefficient under different turn number ratio and duty cycle.

*n* (turn ratio)	*D* (duty ratio)	Current ripple coefficient
2	60%	5.3%
3	50%	1.8%
4	40%	12.3%

**Table 4:** Simulation parameters.

The proposed converter parameters	Value
*V*_in_ (V)	1.3
*n* (turn ratio)	*N*_*s*_/*N*_*p*_ = 1 : 3
*L*_m1_, *L*_m2_ (*μ*H)	7
*C*_1_, *C*_2_, *C*_3_, *C*_4_ (*μ*F)	100
*f*_*s*_ (KHz)	100
*D* (duty ratio cycle)	50%

**Table 5:** Simulation results under seawater battery output conditions.

*V*_in_ (V)	*I*_in_ (A)	Current ripple (A)	*S*_1_, *S*_2_ voltage stress (V)	Duty ratio (%)	*V*_out_ (V)
1.2	8.33	0.31	3.62	55	24
1.25	8.00	0.22	3.54	52	24
1.3	7.69	0.15	3.80	50	24
1.35	7.41	0.18	3.71	45	24
1.4	7.14	0.29	3.76	41	24

**Table 6:** Experimental results under seawater battery output conditions.

*V*_in_ (V)	*I*_in_ (A)	Current ripple (A)	*S*_1_, *S*_2_ voltage stress (V)	Duty ratio (%)	*V*_out_ (V)	Efficiency (%)
1.2	10.7	0.38	3.84	57	23.6	78.2
1.25	10.1	0.27	3.67	53	23.8	79.1
1.3	9.4	0.2	4.00	50	24.0	81.9
1.35	8.9	0.22	3.92	46	24.0	82.5
1.4	8.5	0.34	3.86	43	24.2	84.2

**Table 7:** Theoretical loss value.

Element	Coupled inductance	*D*_1_	*D*_2_	*D*_3_	*D*_4_	*S*_1_, *S*_2_
*P*_loss_ (W)	1.57	0.15	0.21	0.21	0.21	0.24

## Data Availability

The data underlying the results presented in the study are available within the manuscript.
